# The Construction of a Special Physical Quality Evaluation System for Outstanding Chinese Male Boxers

**DOI:** 10.1155/2022/7319602

**Published:** 2022-07-04

**Authors:** Xiangui Bu

**Affiliations:** School of Competitive Sports, Shandong Sport University, Rizhao 276800, China

## Abstract

To construct a structural model of special physical quality test indexes for Chinese outstanding male boxers and to develop comprehensive evaluation criteria for special physical quality of Chinese outstanding male boxers. Expert questionnaire survey method, principal component analysis, and R-type factor analysis were applied in this study. Results of this study include, (1) Through factor analysis, the four types of factors that play a major role for male boxers were strength factor, speed factor, endurance factor, and agility factor in order. (2) Through principal component analysis and R-type factor analysis, the regression equation of the estimated values of the common factors was obtained, and the formula for calculating the comprehensive development level of physical quality of Chinese outstanding male boxers was established through weighting. (3) Through the empirical test, the gap between Level I boxers and boxers at the fitness level was in the endurance and agility dimensions, and Level II boxers were also worse than Level I boxers in the agility dimension, and there was an all-round special physical quality gap between Level II boxers in strength, speed, endurance, and agility and boxers at the fitness level. Conclusion of this study could be summarized as follows: first, the special physical quality index system of Chinese excellent male boxers is: 1 min power sandbag, 20 s straight punch, 9 min double swing jump rope, 1 min front and back hand exchange sandbag 4 items. Second, the standard scores of 4 special physical quality indexes for Chinese outstanding male boxers were developed. Third, the formula for calculating the comprehensive score of special physical quality development level of Chinese excellent male boxers was developed: *T* = ∑*WiTi* = 0.367*T*1 + 0.307*T*2 + 0.172*T*3 + 0.154*T*4. Fourth, the evaluation criteria for the comprehensive physical quality development level of Chinese excellent male boxers were established (*T* ≥ 72.01 for excellent; 44.6 ≤ *T* < 72.01 as good; *T* < 44.6 as poor).

## 1. Introduction

With the promulgation of the new rules of boxing by the International Boxing Federation, boxing matches are becoming more and more intense, and the direct physical confrontation is enhanced, which puts forward higher requirements on the special physical quality of boxers. The situation in the boxing ring is changing rapidly. The athletes have to make judgments and take action in a very short time, using good physical quality, skillful techniques, and variable tactics of attack and defense. High-intensity direct physical confrontation in boxing has high requirements for special speed, strength, endurance, and agility. The construction of a special physical quality evaluation system for excellent male boxers can effectively evaluate the development level of the special physical quality of male boxers and provide a theoretical basis for targeted improvement of special ability training. Therefore, this study draws on advanced training concepts from abroad, combines the physical condition of Chinese male boxers, explores the special physical characteristics of Chinese male boxers, selects special physical indicators for quantitative analysis, and measures and analyzes athletic performance to determine. This study explores the special physical quality characteristics of Chinese male boxers by taking into account the physical conditions of Chinese male boxers.

## 2. Research Subjects and Research Methods

### 2.1. Research Subjects

The Chinese men's boxing training team consisted of 63 individuals, aged (19.2 ± 1.68) years, with a training period of (6.43 ± 2.80) years, including 19 athletes at the fitness level, 24 athletes at the first level, and 20 athletes at the second level.

### 2.2. Research Methods

#### 2.2.1. Expert Interview Method

A total of 26 interviews were conducted with Chinese boxing team coaches and physical fitness experts to propose matters related to the special physical fitness test indexes of Chinese outstanding male boxers and to lay an empirical foundation for the study.

#### 2.2.2. Questionnaire Method

Based on the expert interviews and practice, 17 indicators related to the special physical quality of Chinese outstanding male boxers were selected and questionnaires were conducted. 26 questionnaires were distributed, 25 were recovered, the recovery rate was 96.2%. Of the 23 valid questionnaires, the efficiency rate was 92%.

#### 2.2.3. Testing Method

For the 12 male boxers' special physical quality measurement indexes initially determined, the research subjects were tested on-site based on the development of relevant testing rules.

*(1) Selection of Test Indexes*. After practical observation and experience summary, combined with the characteristics of the boxing project, 17 test indexes were selected for excellent male boxers: (1) strength quality: 20 s barbell bench press (record times), standing triple jump (record distance), 1 min power sandbag (record times), 20 s sit-ups (record times), and 30 m half-squat jump (record distance); (2) speed quality: 10 m × 4 folding run, 20 s straight punch (record times), 20 s swinging punch (record times), and 20 s uppercut (record times); (3) endurance quality: 9 min double punch (record times) , 20 s uppercut (record times), 20 s straight punch (record times), 20 s swinging punch (record times), and 20 s uppercut (record times); (3) endurance quality: 9 min double shake jump rope (record times), 1 min pinch arm push-ups (record times), and 1 min combination pace (record times); (4) sensitivity quality: 1 min front and back hand exchange sandbag (record times), cross quadrant running (record time), and 30 s see signal pace; (5) flexibility quality: left shoulder joint posterior stretch angle (remember the angle) and right shoulder joint posterior stretch angle (remember the angle).

#### 2.2.4. Mathematical and Statistical Method

Descriptive statistics, correlation coefficient method, principal component analysis and factor analysis method, and method of deviation were used to statistically process the raw data by using SPSS 13.0 software.

## 3. Results and Discussion

### 3.1. Review of the Overall Development Level of Boxing in China

The background of China's national system of competitive sports has provided motivational support for the development of boxing, which is highly competitive, less marketable, and less popular. In recent years, with the rising level of China's market economy and the flourishing of professional sports events, the pace of professionalization of boxing in China has accelerated and boxing has received more and more attention in China. However, in terms of the number of registered boxers, there is still a gap between China's 900 registered boxers and more than 8,000 boxers in the Philippines and 16,000 boxers in Japan [1], and the development of boxing in China still lags behind its Asian neighbors, such as Japan and the Philippines, as well as European and American countries.

From Tables 1 and 2, it can be seen that in 2021, among the statistics of the top 10 boxers in the P4P ranking of domestic and foreign professional male boxers, the top P4P ranking of Chinese outstanding male boxers are mostly in the flyweight, featherweight, and lightweight classes, while the middleweight, super middleweight, light heavyweight, and heavyweight classes Chinese male boxers are less, compared with the outstanding male boxers from Europe and America. Due to racial differences Chinese male boxers are at a disadvantage in terms of height, arm span, and weight, and their performance in middle and big level competitions is biased, making it relatively difficult to break through. In addition, from the annual P4P ranking of the top 10 Chinese and foreign male boxers in terms of number of matches and win rate, we can see that the average number of matches of Chinese male boxers is 14.5, which is much lower than the average number of matches of foreign male boxers. The average number of fights per year is much lower than the average of 29.4 fights per year for foreign male boxers. In order to achieve excellent results in professional and amateur boxing, Chinese men's boxing should develop special physical qualities according to their own physical conditions and characteristics, so as to lay a physical foundation for Chinese men's boxing to achieve excellent competition results.

### 3.2. Primary Selection of Special Physical Quality Test Indexes for Chinese Outstanding Male Boxers

Dee Martin believes that special sports qualities refer to the performance of special physical qualities and abilities in sports, and special physical qualities are closely related to special and are physical qualities that can directly promote the mastery of special techniques and improve special performance [2]. Different sports have different requirements for various qualities, and the contribution of various physical qualities to the competitive ability of different sports varies, and only when various qualities play a comprehensive role can we achieve excellent results. According to the item group training theory put forward by Professor Tian Maijiu, boxing is a skill-dominated, same-field combat item group, which requires athletes to be able to maintain sufficient physical energy in continuous multiround direct physical confrontation.

As shown in Table 3, 17 test indexes were selected as the initial indexes for the special physical fitness test of Chinese male boxing athletes, and a questionnaire survey of 26 boxing coaches, sports training experts, and physical training experts was conducted to establish the test index system for the special physical fitness indexes of male boxing athletes. Each index is classified as very important, important, average, unimportant, and unimportant in five levels of influence on the physical quality of boxers, and according to the questionnaire method, the level questions can be measured using the level scale, and in the mathematical and statistical analysis, the numerical values are numerical according to the level “5, 4, 3, 2, and 1” [3]. In the percentage standard, the good standard is 75 points, and according to the percentage calculation standard, the good standard score of each indicator is determined as 3.75 points. After the questionnaire survey, the average value of each grade is obtained, and 12 indicators with a score of 3.75 or more are initially determined (1 means selected, 0 means discarded). The stability and reliability of the 12 test indicators were tested, and the reliability correlation coefficient: *r* = 0.976, *P* < 0.01, and the structural validity correlation coefficient: *r* = 0.918, *P* < 0.01, were tested to be highly significant.

### 3.3. Structural Modeling of Special Physical Quality Test Indexes for Chinese Male Boxing Athletes

#### 3.3.1. Principal Component Analysis of Special Physical Quality Test Indexes for Chinese Male Boxers

According to the principle of statistics, the more test items, the greater the amount of information. However, too many test items will bring difficulties to the test, calculation, and analysis, thus affecting its promotion and application [4]. Boxing special physical fitness test indexes should not only reflect the boxing sport requirements for special physical fitness but also make the test indexes accurately reflect the actual boxing sport items, so as to achieve fewer but more precise. Therefore, the 12 test items need to be screened again to select simple and feasible indicators that are representative of boxing. In order to determine the final test indexes, principal component analysis was used to statistically process the data of the 12 test indexes to obtain the eigenvalues, contribution rates, and cumulative contribution rates of the test sample correlation matrix, and select the principal components with eigenvalues greater than 1 and cumulative contribution rates of 85%, which reflect the special physical fitness level of excellent male boxers (see Table 4). Since the eigenvalue of principal component 5 was 0.98 close to 1, and the cumulative contribution rate of the first five principal components was about 85%, five principal components were selected.

#### 3.3.2. R-Type Factor Analysis of Special Physical Fitness Test Indexes of Chinese Outstanding Male Boxers

According to the number of test index values greater than 1 index, 5 principal components were selected (see Table 5), and the initial factor matrix was rotated by maximum variance to obtain factor loadings on each principal component with larger indexes, and the 5 factors were named according to the original meanings of these variables (see Table 6). After principal component and R-type factor analysis, the 5 categories of factors that play a major role for male boxers are strength factor, speed factor, endurance factor, agility factor, and flexibility factor in order. The physical performance in sports is a combination of various qualities, and a purely physical quality cannot determine whether an athlete's overall physical quality is good or bad. Boxing athletes need to strengthen the comprehensive physical quality training to achieve excellent competition results.

Boxing requires athletes to have good explosive power, very fast punching speed, fast movement, flexible dodging, and long-lasting endurance. According to the principal component analysis and boxing coaches' experience, the flexibility quality is not very important in boxing and does not play a dominant role in winning or losing the match, so the requirements are relatively low and can be ignored in the test. So, strength, speed, endurance, and agility are especially important for boxers.

Strength is the basis for participation in all sports and poor strength quality will limit the development of other qualities. Boxing is a competitive game of close combat in which the opponent is won by a quick blow to the effective part of the body or by a heavy knockout punch. With the promulgation of the new rules of boxing, the physical confrontation of boxing is more intense, heavy punches can effectively hit the opponent hard or directly end the game, power quality is the basis of boxing heavy punches, so the greater the power, the greater the striking force on the opponent, the stronger the killing force; conversely, the smaller the power, the smaller the striking force on the opponent, not only cannot effectively hit the opponent but also by the opponent to grab the first opportunity, and thus in a passive position. That is why strength is the first factor to win a boxing match.

According to the principles of physics, momentum is a physical quantity related to the mass and velocity of an object, expressed by the formula: *P*=*m* − *v*, with *P* being momentum, *m* being mass, and *v* being velocity. The speed of the punch is crucial for boxers of the same level to obtain a large momentum. Fast punches in boxing can effectively destroy the opponent's offensive intentions and at the same time can pre-emptively strike the opponent, interfere with the opponent's offensive distance, and create the time for their heavy punches to hit. In addition, boxing requires a flexible pace and fast and slow foot movement, which is important for the articulation of technical movements and tactical use. Therefore, boxers should improve their punching speed and movement speed on top of increasing their strength [5]. So speed is the second factor that should be focused on developing.

In amateur and professional boxing matches, there are 3 rounds, 6 rounds, 8 rounds, 10 rounds, and 12 rounds of different systems, with a 1 minute rest in the middle of the rounds, which puts high demands on the quality of endurance. In boxing, due to the long competition time, endurance plays a role in guaranteeing the technical and tactical level. If the athletes have better endurance reserves, then the athletes' technical and tactical implementation will be more resolute, without the worry of physical fitness. From the viewpoint of energy consumption, boxing is mainly supplied by the ATP-CP system and anaerobic enzyme system, which have a relatively short maintenance time, while the metabolites of the anaerobic enzyme system, lactic acid, are difficult to clear in a short time, which will cause boxers' muscles to be sore and swollen, and the excitability of the nervous system to be reduced, manifesting as slower punching speed, weaker power, and slower reaction. If boxers do not have good endurance quality, their skills and tactics will not play properly. Endurance quality as is the third factor affecting their competitive ability.

Boxing allows striking and scoring parts to be head and face, neck, chest, both ribs, and small abdomen, and athletes should avoid being hit by opponents in effective scoring parts during the game, so flexible dodging and foot movement, along with good body control, are the main technical means to avoid being hit by opponents [6]. Boxing in the game of offense and defense is relatively fast, especially for the best athletes, so the body's sensitive quality is an indispensable component of effective defense. A variety of offensive and defensive actions need to be coordinated with the body of punches and feet to complete the action, for the control of the opponent's attack distance and destroying the opponent's rhythm has an important role. The four categories of boxer physical fitness factors have different effects on the athletic ability of athletes, but combined, they are indispensable for the improvement of the athletic ability of boxers.

The regression equation of the common factor estimates was calculated by principal component analysis and R-type factor analysis:

 
*Z*1 = 0.68*X*1 + 0.46*X*2 + 0.64*X*3 + 0.24*X*4 + 0.62*X*5 + 0.36*X*6 + 0.28*X*7 + 0.42*X*8 + 0.33*X*9 + 0.31*X*10 + 0.23*X*11 + 0.25*X*12.
 
*Z*2 = − 0.56*X*1 − 0.52*X*2 − 0.39*X*3 − 0.74*X*4 − 0.48*X*5 + 0.26*X*6 − 0.72*X*7 − 0.42*X*8 − 0.63*X*9 + 0.41*X*10 – 0.23*X*11 + 0.22*X*12.
 
*Z*3 = 0.68*X*1 + 0.46*X*2 + 0.34*X*3 + 0.44*X*4 + 0.32*X*5 + 0.16*X*6 + 0.20*X*7 + 0.74*X*8 + 0.76*X*9 + 0.31*X*10 + 0.25*X*11 + 0.19*X*12.
 
*Z*4 = 0.43*X*1 + 0.67*X*2 + 0.32*X*3 + 0.34*X*4 + 0.32*X*5 + 0.12*X*6 + 0.24*X*7 + 0.42*X*8 + 0.46*X*9 + 0.51*X*10 + 0.69*X*11 + 0.14*X*12.

The standardized values of the 12 quality indicators were substituted into the equation to obtain the common factor estimates, which were used to judge and analyze the individual quality characteristics of boxers and conduct targeted training. Meanwhile, the sum of the four factor scores could also evaluate the special physical quality training level of boxers at the same level. From the results of factor analysis, the development of the special physical quality of excellent male boxers shows multiple aspects, so the evaluation of their special physical quality should be carried out for the four categories of indicators derived from factor analysis, and the principal components involve a large number of their special physical test indicators, so 1–2 indicators from each principal component can be selected as representatives according to the factor loading size to determine the typical test indicators of each category.

The first principal component, 1 min strength sandbag, is the boxer's upper limb explosive strength index, and 30 m semisquat jump is the lower limb explosive strength index. The 1 min power sandbag is the largest load, so the 1 min power sandbag (*Y*1) is chosen as the representative index.

The second principal component, 20 s straight punch, 20 s swinging punch, and 10 m × 4 folding run are important indicators of boxers' punching speed and moving speed. 20 s straight punch (*Y*2) has the largest load and is often used in boxing special training, so 20 s straight punch is chosen as a representative indicator.

The third principal component, 1 min arm clamping push-ups, followed by 9 min double rocking jump rope testing boxers' upper and lower limb endurance, is an important indicator to measure their upper and lower limb endurance. 9 min double rocking jump rope load is the largest time in line with the boxing competition time requirements, so choose the 9 min double rocking jump rope (*Y*3) as a representative index.

The fourth principal component, 1 min front and back hand exchange sandbag, 30 s look at the signal pace movement, is an important index of boxers' sensitivity quality. The boxing match is at least 3 rounds system, more than 12 rounds system, and high intensity fighting confrontation in the endurance quality puts forward high requirements. 1 min front and back hand exchange sandbag load is larger, choose the 1 min front and back hand exchange sandbag (*Y*4) as the endurance quality index.

### 3.4. Development of Comprehensive Evaluation Criteria for Special Physical Quality of Chinese Outstanding Male Boxers

#### 3.4.1. Development of the Rating Scale for Each Test Index of the Special Physical Quality of Male Boxers

As shown in Table 7, since the measurement indexes of male boxers are tested with different measurement units, the evaluation methods and standards are different, which is not easy to calculate, analyze, and compare, and if the measurement results are used directly, it cannot accurately evaluate the special physical quality of boxers comprehensively, so it is necessary to standardize the evaluation indexes and convert the measured values of the special physical quality test indexes into unified measurement parameters for comprehensive evaluation. Therefore, it is necessary to standardize the evaluation indexes and transform the measured values of each special physical fitness test index into a unified metric in order to make a comprehensive evaluation. In this study, the mean was used as the benchmark, and the standard deviation was used as the discrete distance to calculate the scores of the indexes and arrange them in an orderly manner, so as to develop the scoring table of each individual special physical quality index.

From Table 7, it can be seen that the larger the *T* value, the higher the overall comprehensive level of special physical fitness of male boxers, and the corresponding higher their comprehensive competitive ability.

#### 3.4.2. Establishment of a Weighted Formula for Calculating the Special Physical Quality of Chinese Outstanding Male Boxers

In order to better reflect the importance of the evaluation indexes of the special physical quality of male boxers, this study adopts the weighting method, which means that each index is weighted according to its importance. The weighting coefficients were determined by dividing the eigenvalues of each evaluation index in the principal component analysis by the sum of the eigenvalues of the four principal components, respectively, to obtain the ranking of the weighting coefficients of each index (see Table 8). According to the analysis of the results in Table 8: 1 min power sandbag weight coefficient is the largest, 0.367, boxing physical combat confrontation project characteristics, absolute power is to complete the boxing technical action guarantee; 20s straight punch weight coefficient is 0.307, is to reflect the speed of punching test index, boxing game offensive and defensive transition speed is very fast, offensive punching and defensive technology conversion instantly completed, so the boxer The speed of action is high [7]; 9 min double shaking jump rope is an important index reflecting the special endurance quality, the weighting coefficient is 0.172, boxing match at least 3 rounds system, has high requirements for endurance quality; 1 min front and back hand exchange sandbag is an important reflection of the sensitivity quality, the weighting coefficient is 0.154.

The formula for calculating the comprehensive development level of physical fitness of outstanding Chinese male boxers is *T* = ∑*WiTi* = 0.367*T*1 + 0.307*T*2 + 0.172*T*3 + 0.154*T*4, Where, *T* denotes the standard score of comprehensive development level of physical quality; Wi denotes the weight value of each special index; Ti denotes the standard percentage obtained from the special index (see Table 7 for the standard percentage comparison table).

#### 3.4.3. Development of Evaluation Criteria for the Comprehensive Development Level of Special Physical Quality of Chinese Outstanding Male Boxers

Sports practice proves that the higher the level of comprehensive development of physical fitness, the stronger the material basis for mastering and improving techniques and tactics, and the greater the potential for improving athletic ability of athletes [8]. According to the principle of normal distribution, when the number of samples is greater than 50, the results of the comprehensive development level of special physical fitness of male boxers can be approximated as obeying normal distribution. According to the principle of 3*σ* (*σ* is the variance), in the normal distribution, *μ* ± 3*σ* contains 99.73% of the information of the variable (*μ* is the mean), so we can find the variance and mean of the sample, and judge the male boxers' performance as excellent if it is higher than *μ* + 1.5*σ*; judge the male boxers' performance as good if it is between *μ* *−* 1.5*σ* and *μ* + 1.5*σ*; judge the male boxers' performance as good if it is lower than *μ* *−* 1.5*σ*; judge the male boxers' performance as good if it is lower than *μ* *−* 1.5*σ*. athletes with scores below *μ* *−* 1.5*σ* were judged as poor (see Figure 1).

The results showed that 13% of the athletes had excellent criteria, and the evaluation criteria were divided into 3 levels of excellent, good and poor according to the distribution of performance to divide the comprehensive evaluation criteria results (see Table 9).

#### 3.4.4. Empirical Analysis of Special Physical Fitness Test Indexes of Chinese Outstanding Male Boxers

Analysis of variance (ANOVA), also known as *F*-test, is used to test the significance of the difference between the means of two and more samples. According to the four test indicators between the different male boxers tested to assess the differences between their strength, speed, endurance and sensitivity, according to Table 10 significant *P* values are less than 0.05, it can be seen that within the 95% confidence interval boxers of the fitness level have a significant difference with the first-class boxers and second-class boxers in general between strength, speed, endurance, and sensitivity.

ANOVA alone can only determine the variability between the totals, while using the LSD multiple comparison method, it is possible to test whether there is a significant difference between the sample means after ANOVA. The data in Table 11 show that in terms of strength and speed, the *P* values of boxers at the fitness level and boxers at the first level are greater than 0.05, which means that there is no significant difference between them in terms of strength and speed. The *P* value between the two and the second level athletes is less than 0.05, which shows that the second level athletes are inferior to the generalist and first level athletes in terms of the factors that contribute most to their performance, so the second level boxers need to strengthen their strength and speed training in order to improve their overall competitive ability. Boxing is a combination of punching, dodging, and pace, and it is important to maintain good endurance and agility during the competition, and to seize the opportunity to deliver a fatal blow to the opponent at the critical moment, which is the main aspect that differentiates the boxers of the first and second levels.

In general, the gap between the first level boxers and the general boxers is in endurance and agility, the second level boxers are also inferior to the first level boxers in this regard, and the second level boxers have a full range of special physical quality gap in strength, speed, endurance, agility, and general boxers.

## 4. Conclusion

1. Based on the expert survey, the statistical quantitative analysis method was used to determine the special physical quality index system of Chinese excellent male boxers: 1 min power sandbag, 20 s straight punch, 9 min double shake jump rope, and 1 min front and back hand exchange sandbag 4 items, which can reflect the special physical quality of Chinese excellent male boxers more objectively.
2. The standard scores of 4 special physical quality indexes of Chinese excellent male boxers were developed by using the method of deviation.
3. Using principal component analysis and R-type factor analysis, the original data were processed to obtain the characteristic values of the 4 test indicators, the weight coefficients of each test indicator, and the formula for calculating the comprehensive score of the special physical quality development level of Chinese excellent male boxers was formulated: *T* = ∑*WiTi* = 0.367*T*1 + 0.307*T*2 + 0.172*T*3 + 0.154*T*4.
4. The evaluation criteria of the comprehensive physical quality development level of Chinese outstanding male boxers were established according to the normal distribution characteristics (*T* ≥ 72.01 was excellent; 44.6 ≤ *T* < 72.01 was good; *T* < 44.6 was poor), and one-way ANOVA and LSD multiple comparisons were applied to derive the variability among boxers of different levels in strength, speed, endurance, and sensitivity.

## Figures and Tables

**Figure 1:** Normal distribution of the overall performance of Chinese outstanding male boxers.

**Table 1:** P4P ranking and physical condition of outstanding Chinese professional male boxers in 2021.

Ranking	Name	Height (cm)	Arm span (cm)	Level	Winning percentage
1	Cao Xingru	170	177	WBO super flyweight	22-0
2	Xu Can	175	175	WBA super featherweight	13-2
3	Ge Wenfeng	165	165	WBO super flyweight	10-0
4	Xiong Chaozhong	155	160	WBA mini lightweight	27-7-1
5	Zou Shiming	162	164	WBO flyweight	9-2
6	Zhang Zhilei	201	210	WBO heavyweight	18-0
7	Baisanbo	180	181	WBC super lightweight	12-1-1
8	Meng Fanlong	190	190	WBO light heavyweight	12-0
9	Sun Xuanxiang	170	170	WBO lightweight	12-0
10	Wang Zhimin	174	173	WBC super lightweight	10-2

Data source: boxing voyager https://www.qjhm.net.

**Table 2:** P4P ranking and physical condition of outstanding foreign professional male boxers in 2021.

Ranking	Name	Height (cm)	Arm span (cm)	Level	Winning percentage
1	Gennady Golovkin	179	178	WBC/WBA/IBF/IBO middleweight	37-0-1
2	Trens Crawford	173	178	WBC/WBO ultra-lightweight	32-0
3	Vassel Lomachenko	168	166	WBO bantamweight	10-1
4	Sergey Kovalev	183	184	WBO lightweight	31-2-1
5	Saul Avarez	175	180	WBO super middleweight	49-1-2
6	Mickey Garcia	168	173	WBC lightweight	37-0
7	Shoya Inoue	162	172	WBO super flyweight	15-0
8	Errol Spence Jr.	177	183	IBF welterweight	22-0
9	Guremo Rigondeaux	164	168	WBA ultra-lightest weight	17-1
10	Srisaket	160	162	WBC ultra-lightweight	44-4-1

Data source: boxing voyager https://www.qjhm.net.

**Table 3:** China's outstanding male boxers special physical fitness test index survey table.

Specialized physical fitness indicators	Score	Selection status
9 min double shake jump rope (record times)	4.22	1
Standing triple jump (remember the distance)	3.43	0
10 m × 4 folding run (record time)	4.78	1
20 s sit-ups (remember the number of times)	3.57	0
Posterior extension angle of the right shoulder joint (remember the angle)	3.91	1
1 min power sandbag (record times)	4.04	1
1 min pinch arm push-ups (record times)	3.91	1
20 s swing (remember the number of times)	4.30	1
20 s uppercut (remember the number of times)	3.57	0
Left shoulder joint posterior extension angle (remember the angle)	4.17	1
1 min combination pace (record times)	3.22	0
1 min front and back hand exchange sandbag (record times)	4.13	1
20 s straight punch (remember the number of times)	4.65	1
Cross quadrant run (keep track of time)	2.74	0
30 s to see the signal pace moving	4.17	1
30 m half squat jump (remember the distance)	4.00	1
20 s barbell bench press (remember the number of times)	4.30	1

**Table 4:** Principal component analysis of special physical fitness test indexes of Chinese outstanding male boxers.

Principal components (indicators)	Eigenvalue	Contribution rate (%)	Cumulative contribution rate (%)
1	3.45	28.1	28.1
2	2.89	23.5	51.6
3	1.62	13.2	64.8
4	1.45	11.8	76.6
5	0.98	8.0	84.5
6	0.51	4.1	88.7
7	0.35	2.8	91.5
8	0.31	2.5	94.1
9	0.24	2.0	96.0
10	0.22	1.8	97.8
11	0.16	1.3	99.1
12	0.11	0.9	100.0

**Table 5:** Matrix of loading factors after great orthogonal rotation of special physical fitness test indexes of Chinese outstanding male boxers.

Indicators	Factor1	Factor2	Factor3	Factor4	Factor5
30 m half squat jump (*X*1)	0.85				
30 s look at the signal pace of movement (*X*2)				0.46	
20 s barbell bench press (*X*3)	0.34				
20 s straight punch (*X*4)		−0.85			
1 min power sandbag (*X*5)	0.87				
Left shoulder joint posterior extension angle (*X*6)					0.65
20 s pendulum (*X*7)		−0.76			
1 min pinch arm push-ups (*X*8)			0.54		
9 min double swing jump rope (*X*9)			0.69		
10 m × 4 folding run (*X*10)		0.69			
1 min front and back hand exchange sandbag (*X*11)				0.58	
Right shoulder joint posterior extension angle (*X*12)					0.73

**Table 6:** Classification and naming of principal components of special physical fitness test indexes of Chinese outstanding male boxers.

Principal components	High load index	Factor naming
1	1 min power sandbag, 30 m half squat jump, 20 s barbell bench press	Strength factor
2	10 m × 4 folding run, 20 s straight punch, 20 s swinging punch	Speed factor
3	1 min clip arm push-ups, 9 min double swing jump rope	Endurance factor
4	1 min front and back hand exchange sandbag, 30 s see the signal pace of movement	Sensitivity factor
5	Left shoulder joint posterior extension angle, right shoulder joint posterior extension angle	Flexibility factor

**Table 7:** Standard scores of special physical fitness test indicators for Chinese outstanding male boxers.

*T*	*Y*1	*Y*2	*Y*3	*Y*4
100	80.42	141.29	901.25	65.14
95	78.13	136.73	883.34	63.48
90	75.86	132.21	860.46	61.32
85	71.24	127.65	835.57	59.46
80	69.34	122.32	817.69	57.35
75	66.85	119.98	791.93	55.79
70	64.27	116.66	765.43	53.38
65	61.75	113.01	744.26	52.41
60	58.99	110.79	726.1	50.57
55	57.48	106.84	702.48	48.93
50	55.1	103.53	674.32	47.02
45	52.92	98.26	654.67	45.28
40	49.23	95.19	631.8	43.71
35	47.97	91.65	608.33	42.99
30	45.36	87.28	584.76	40.17
25	42.18	83.46	562.49	38.63
20	39.87	79.32	538.04	37.02
15	37.45	75.32	516.97	36.87
10	34.9	71.04	493.23	33.54
5	31.71	66.38	473.46	31.73
0	29.68	62.41	447.35	30.12

**Table 8:** Table of weighting values of special physical fitness test indicators for Chinese outstanding male boxers.

Indicators	*Y*1	*Y*2	*Y*3	*Y*4
Weights	0.367	0.307	0.172	0.154
Sort by	1	2	3	4

**Table 9:** Excellent boxers special physical quality comprehensive evaluation criteria table.

Grade	Standard
Excellent	*T* ≥ 72.01
Good	44.6 ≤ *T* < 72.01
Poor	*T* < 44.6

**Table 10:** One-way ANOVA of special physical fitness test indexes of Chinese outstanding male boxers.

		Sum of squares	Degrees of freedom	Mean square	*F*	Significance *P*
Strength	Intergroup	1725.888	2	862.944	51.247	0.000
	Within groups	1010.334	60	16.839		
	Total	2736.222	62			

Speed	Intergroup	2452.074	2	1226.037	16.622	0.000
	Within groups	4425.672	60	73.761		
	Total	6877.746	62			

Endurance	Intergroup	64906.636	2	32453.318	12.662	0.000
	Within groups	153782.221	60	2563.037		
	Total	218688.857	62			

Sensitive	Intergroup	437.353	2	218.676	19.477	0.000
	Within groups	673.631	60	11.227		
	Total	1110.984	62			

**Table 11:** LSD multiple comparison table of special physical fitness test indexes of outstanding male boxers.

Dependent variable			Average difference	Standard error	Significance *P*	95% confidence interval	
						Lower limit value	Upper limit
Strength	Fitness level	Level 1	9.382^*∗*^	1.817	0.000	5.75	13.02
		Level 2	17.326^*∗*^	1.881	0.000	13.56	21.09
	Level 1	Fitness level	−9.382^*∗*^	1.817	0.000	−13.02	−5.75
		Level 2	7.944^*∗*^	1.108	0.000	5.73	10.16
	Level 2	Fitness level	−17.326^*∗*^	1.881	0.000	−21.09	−13.56
		Level 1	−7.944^*∗*^	1.108	0.000	−10.16	−5.73

Speed	Fitness level	Level 1	4.892	3.803	0.203	−2.72	12.50
		Level 2	16.790^*∗*^	3.937	0.000	8.91	24.67
	Level 1	Fitness level	−4.892	3.803	0.203	−12.50	2.72
		Level 2	11.898^*∗*^	2.319	0.000	7.26	16.54
	Level 2	Fitness level	−16.790^*∗*^	3.937	0.000	−24.67	−8.91
		Level 1	−11.898^*∗*^	2.319	0.000	−16.54	−7.26

Endurance	Fitness level	Level 1	−0.147	22.418	0.995	−44.99	44.70
		Level 2	66.543^*∗*^	23.208	0.003	20.12	112.97
	Level 1	Fitness level	0.147	22.418	0.995	−44.70	44.99
		Level 2	66.691^*∗*^	13.668	0.000	39.35	94.03
	Level 2	Fitness level	−66.543^*∗*^	23.208	0.003	−112.97	−20.12
		Level 1	−66.691^*∗*^	13.668	0.000	−94.03	−39.35

Sensitive	Fitness level	Level 1	6.127^*∗*^	1.484	0.000	3.16	9.10
		Level 2	9.312^*∗*^	1.536	0.000	6.24	12.38
	Level 1	Fitness level	−6.127^*∗*^	1.484	0.000	−9.10	−3.16
		Level 2	3.184^*∗*^	0.905	0.001	1.37	4.99
	Level 2	Fitness level	−9.312^*∗*^	1.536	0.000	−12.38	−6.24
		Level 1	−3.184^*∗*^	0.905	0.001	−4.99	−1.37

## Data Availability

All data used in this study can be accessed upon reasonable request to the author.
